RETRACTED

# Correlation Analysis of Ultrasound Elastography Score with Invasive Breast Cancer and Biological Prognostic Factors

**DOI:** 10.1155/2022/1174541

**Published:** 2022-07-04

**Authors:** Q. Fu, F. Wan, Q. Lu, W. Shao, G. Fu, Z. Wang

**Affiliations:** ^1^Department of Ultrasound, The Second Hospital of Wuxi Affiliated to Nanjing Medical University, Wuxi 214002, Jiangsu, China; ^2^Department of Ultrasound, The Affiliated Huai'an Hospital of Xuzhou Medical University and the Second People's Hospital of Huai'an, Huai'an 223001, Jiangsu, China

## Abstract

Invasive breast cancer (IBC) is a kind of malignant tumor in which cancer cells have broken through the basement membrane of breast ducts or lobular acini and invaded the stroma. Although ultrasound elastography score (UES) has shown unique advantages in the diagnosis of IBC, its value in the prognosis is not clear. Here, we explored the correlation of UES with IBC and biological prognostic factors. The datum of 86 patients with suspected IBC from January 2018 to December 2021 was collected. UE was applied in the examination of all patients. The lesion tissue of the malignant group was punctured to detect and analyze the expression of biological prognostic factors, including estrogen receptor (E receptor), progesterone receptor (P receptor), and human epidermal growth factor 2 (HER factor 2) and Ki67. The differences in UES under different biological prognostic factors were compared. The receiver operating characteristic (ROC) curve was applied to analyze the diagnostic value of UES of IBC and the expression of biological prognostic factors. Based on the pathological diagnosis results, the sensitivity, specificity, accuracy, positive predictive value, and negative predictive value of UES in the diagnosis of IBC were analyzed. The correlation of UES with IBC and biological prognostic factors was analyzed by multiple linear regression and Spearman method. ROC analysis showed that the area under the curve of UES for diagnosing IBC and evaluating the expression of P receptor, HER factor 2, and Ki67 were 0.877, 0.704, 0.763, and 0.820, respectively (*P*＜0.05). The sensitivity, specificity, accuracy, positive predictive value, and negative predictive value of UES when diagnosing IBC were 92.42%, 90.00%, 91.86%, 96.83%, and 78.26%, respectively. The UES of *E* receptor expression (positive and negative group) showed no obvious variance (*P* > 0.05). The UES of P receptors (positive and negative), HER factor 2 (positive and negative), and Ki67 (high and low expression) showed obvious differences (*P* < 0.05). Multiple linear regression and Spearman indicated UES was significantly correlated with the expression of P receptor, HER factor 2, and Ki67 (*P*＜0.05). UES has a certain diagnostic value for IBC and is significantly correlated to the expression of P receptor, HER factor 2, and Ki67, which is helpful for evaluating the prognosis of patients with IBC.

RETRACTED

## 1. Introduction

Breast cancer is the most common malignant tumor in women. Invasive breast cancer (IBC), the most common type of breast cancer, refers to a malignant tumor in which cancer cells could penetrate into the basement membrane of breast ducts or lobular acini. The incidence rate and the mortality rate of breast cancer ranked first and fourth among female malignant tumors in China. In 2016, there were about 290,500 cases of female breast cancer in China, accounting for 17.1% of all female malignant tumors. And there were about 63,900 deaths, accounting for 8.2% of all female malignant tumor deaths [1]. With the acceleration of population aging, industrialization, urbanization, and lifestyle changes, the disease burden of female breast cancer is increasing. Improving the detection rate of early breast cancer and timely and effective treatment are effective measures to reduce the mortality of breast cancer. However, breast cancer is prone to missed diagnosis and misdiagnosis, since the early symptoms and signs are mostly inconspicuous and difficult to attract attention [2, 3]. The disease has a different prognosis according to the type of pathological tissue and degree of malignancy. As a result, it is important to find a method to evaluate the prognosis of patients with IBC quickly and effectively [4, 5].

Estrogen receptor (E receptor), progesterone receptor (P receptor), human epidermal growth factor 2 (HER factor (2), and Ki67 are common biological factors related to the prognosis of IBC. *E* receptors and P receptors are a family of steroid hormones that regulate the transcription of target genes after binding to receptors and can promote malignant breast hyperplasia [6]. HER factor 2 can induce the increase of vascular endothelial growth factor in the body, furthermore promoting the formation of tumor angiogenesis, and is closely related to tumor proliferation, invasion, and metastasis [7]. Ki67 is a nuclear antigen associated with proliferating cells and closely related to mitosis. It is an important cytokine in cell proliferation. Ki67 is related to the degree of malignancy, active proliferation, growth rate, and probability of lymph node metastasis and expressed at high levels in the proliferation stage of the tumor [8, 9]. However, the detection of the above factors relies on needle biopsy, which is often inconvenient. Ultrasound elastography (UE) is a new-emerging ultrasound diagnostic technology, used for detecting diffuse diseases in a simple and quick manner instead of traditional ultrasound imaging [10, 11].

RETRACTED

In the context of the above research, this study retrospectively analyzed the correlation of ultrasound elastography score (UES) with IBC and biological prognostic factors, in order to lay the foundation for preventing and treating IBC.

## 2. Materials and Methods

### 2.1. General Data

The datum of 86 patients with suspected IBC from Jan 2018 to Dec 2021 was chosen for the present research. According to the pathological diagnosis results [12], 66 and 20 patients were malignant and benign, respectively. This study was approved by the meeting of the Medical Ethics Committee of our hospital, and all examinations were obtained with the informed consent of the patients.

Inclusion criteria:

1. Patient with suspected IBC diagnosed by clinical and imaging examinations
2. Patients without tumor surgery, radiotherapy and chemotherapy

Exclusion criteria:

1. Patients with tumors in other tissues and organs
2. Patients with contraindications to puncture
3. Pregnant women
4. Patients who cannot cooperate with the examination
5. Patients with incomplete clinical case data

### 2.2. Methods

#### 2.2.1. The Diagnosis of IBC by UE

The color ultrasound diagnostic instrument (Instruments: GE LOGIOE9, Vinno G86) with high-frequency probes was used to conduct longitudinal, lateral and oblique exploration of all lesion areas. The probe frequency is set to 5–15 MHz. Firstly, we use the conventional ultrasound mode to detect the size, shape, echo and the blood supply of the lesion. Secondly, the real-time double-amplitude mode of elastography program is used. The quality factor of the quality control parameters shown on the screen should be greater than or equal to 60, and the sampling frame is adjusted to contain breast mass and the surrounding normal tissue. The region of interest should be located in the center of the sampling frame as much as possible. In the UE system, the tissue with small elasticity will change greatly after being compressed and will turn red, otherwise the tissues will be blue. The modified UE 5-point method [13] was used to evaluate the benign and malignant lesions of suspected lesions: the overall or large area of the lesion was green = 1 point: the central area and surrounding area were blue and green, = 2 points: the inner area of the lesion was blue = 3 points: the area ratio of green and white was close to 1 : 1 = 4 points: the lesion is blue as a whole, or with a little green area scattered inside = 5 points: the lesion area and surrounding are blue, with or without green area inside =, respectively.

#### 2.2.2. Detection of Biological Prognostic Factors

The tissue material collected by puncture was placed in citrate buffer (0.01 mmol/L) with a pH of 6.0, and heated at 96°C for 10 min. After culturing for 30 min, diaminobenzidine (DAB, Shanghai Yiji) was used as the first antibody and incubated overnight at 4°C. Then, *E* receptor, P receptor, HER factor 2, and Ki67 were added as secondary antibodies and incubated at room temperature for 60 min. At the end, the nuclei were counterstained with hematoxylin and mounted with DAB. Interpretation criteria [14, 15] tumor cell nuclei with brownish-yellow granules accounted for ≥10% were recorded as a positive expression of P receptor and *E* receptor; positive staining cells accounted for ≥14% were recorded as high expression of Ki67 antigen, otherwise, it was recorded as low expression of Ki67 antigen; cell membrane molecules stained at a different level were recorded as 0, +, ++ and +++, among which 0 and<puncsp> </puncsp>+<puncsp> </puncsp>are recorded as HER factor 2 negative, +++ is recorded as HER factor 2 positive, ++ requires, respectively further in situ hybridization gene amplification verification.

RETRACTED

### 2.3. Observation Indicators

1. To analyze the diagnostic value of UES for IBC, and to analyze the sensitivity, specificity, accuracy, and positivity of the UES in the diagnosis of IBC according to pathological diagnosis results.
2. To compare the differences of UES under different expressions of biological prognostic factors, and to analyze the evaluation value of UES for the expression of biological prognostic factors in IBC.
3. To analyze the correlation between the UES and an expression of biological prognostic factors in patients with IBC.

### 2.4. Statistical Methods

Statistical analysis was performed by SPSS 22.0 (IBM Corp, Armonk, NYUSA). Measurement data are represented by mean ± SD, and *t*-test is used for comparison; count data is represented by *n*, and *χ*^2^ test is used for comparison. The receiver operating characteristic (ROC) curve was applied in analyzing UES diagnostic value and evaluation value for biological prognostic factor expression [16]. The area under the curve (AUC) and the 95% confidence interval were calculated, and the cut-off point value was taken as the corresponding value of the cut-off point corresponding to the maximum Youden index (sensitivity + specificity-1). The correlation of UES with IBC and biological prognostic factors was analyzed by multiple linear regressions and Spearman-method. Differences were considered obvious at *P* < 0.05.

## 3. Result

### 3.1. ROC Analysis of UES in the Diagnosis of IBC

ROC analysis shows that the AUC of UE and cut-off value score in the diagnosis of IBC was 0.877 (95%  CI:0.721–0.863) and 3.98, respectively (*P* ＜ 0.05), as shown in Figure 1.

RETRACTED

### 3.2. Diagnostic Value of UES for IBC

Taking pathological diagnosis as the gold standard and referring to cut-off value of the ROC analysis, the sensitivity, specificity, accuracy, positive predictive value, and negative predictive value of the UES in diagnosis of IBC were 92.42%, 90.00%, 91.86%, 96.83% and 78.26%, respectively, as shows in Table 1.

### 3.3. Univariate Analysis of the Correlation

No obvious difference is observed in UES between the *E* receptor negative group and positive group (*P* > 0.05). Nevertheless, P receptor, HER factor 2 and Ki67 are significantly correlated to UES (*P* ＜ 0.05). See Table 2.

### 3.4. ROC Analysis of UES

ROC analysis in Table 3 shows that the AUC of the UES is used for evaluating the expression of P receptor, HER factor 2 and Ki67 were 0.704 (95%  CI:0.600–0.795), 0.763 (95%  CI:0.663–0.845) and 0.820 (95%  CI:0.726–0.893), respectively, as shown in Table 3 and Figure 2.

### 3.5. Correlation Analysis between UES and Biological Prognostic Factor Expression

Taking the statistically significant indicators in Table 2 as independent variables and the UES as the dependent variable, multiple linear regressions analysis and Spearman correlation analysis were performed. UES was significantly correlated with the expression of P receptor, HER factor 2 and Ki67 (*β*/*r* = 0.344/0.238; 0.375/0.295; 0.315/0.334, *P* ＜ 0.05). See Table 4 and 5.

### 3.6. Typical Case

The ultrasound images of a female patient histopathologically diagnosed with the invasive carcinoma were shown as typical case in Figure 3.

Figures 3(a)to 3(d) show a female patient, aged 59, presented with a breast lump, and histopathologically diagnosed with invasive carcinoma after surgical resection.

## 4. Discussion

IBC is a common type with a high degree of malignancy, threatening women's life and health [17]. At present, there are many studies on breast cancer, but its specific etiology is still unknown. In recent years, studies on cancer related biological genes and immunohistochemistry suggested that the occurrence of canceration often causes abnormal changes in some biological factors in the body [18]. These biological factors are often closely related to the prognosis of the disease. At the same time, the inflammatory factors caused by canceration, abnormal expression of tumor cytokines and other factors will further stimulate the proliferation of cancer cells [19]. The analysis of biological prognostic factors related to cancer can provide important guidance for early development of an effective treatment plans for patients with this disease and improvement of patient prognosis. However, the cumbersome procedures and a high cost of biochemical indicator detecting limit its clinical application. As a new-emerging imaging technology, UE is expected to change this situation. This study attempted to correlate the UES with biological prognostic factors and IBC.

RETRACTED

ROC analysis indicated the AUC of the UES for the diagnosis of IBC was 0.877. The sensitivity, specificity, accuracy, positive predictive value, and negative predictive value of UES for diagnosing IBC were 92.42%, 90.00%, 91.86%, 96.83%, and 78.26%, respectively, indicating that the UES has a certain diagnostic value for IBC. To explore the correlation, studies have shown that benign and malignant breast tumors are closely related to tissue hardness. The hardness of malignant tumor lesions is about 2–3 times that of benign tumor lesions. UE provides a specific stimulus to a specific examination site, and the target site produces different bioelastic responses under the stimulus. Malignant masses are hard in texture and have a low elastic deformation ability [20], so malignant masses and benign masses would show a high and a low UES, respectively. UE can objectively reflect the tissue density of the lesions and further identify whether the tissue is malignant.

In this study, we investigated the effect of the UE on factors related to *E* receptor, P receptor, HER factor 2, and Ki67 in breast cancer patients. For *E* receptor and P receptor, they are glycoproteins contained in normal breast epithelial cells, which can bind to estrogen and progesterone, respectively. After the occurrence of breast cancer, some breast cancer can retain all or part of hormone receptors. This kind of breast cancer can be regulated by hormones and is sensitive to endocrine therapy. Some breast cancer may lose all or part of its hormone receptors, which is ineffective for endocrine therapy [21, 22]. Therefore, *E* receptor and P receptor are very important biological indicators of breast cancer. HER-2 protein is a transmembrane glycoprotein, which plays an important role in the process of cell proliferation, differentiation, and angiogenesis [23]. This high expression can accelerate cell division, make the process of proliferation and differentiation unbalanced, and finally turn into cancer cells. About 20% of primary breast cancer have HER-2 gene amplification or protein over expression. Therefore, the expression of HER-2 is very important for judging the diagnosis and treatment of breast cancer patients, and is an important predictor of the effect of chemotherapy and endocrine therapy in breast cancer patients. Ki67 is an index reflecting cell proliferation. Patients with breast cancer often classify molecular subtypes according to the proliferation ratio of Ki67 [24]. For patients with high expression of Ki67, tumor cells often proliferate faster, the degree of malignancy is higher, and the prognosis is often poor. For patients with low expression of Ki67, the prognosis is often better.

RETRACTED

We found that the AUC for evaluating the expression of P receptor, HER factor 2, and Ki67 by UE were 0.704, 0.763, and 0.820, respectively. The UES of P receptor (positive and negative group), HER factor 2 (positive and negative group) and Ki67 (high and low expression group) showed significant difference. Multiple linear regressions and Spearman indicated the UES were significantly correlated with the expression of P receptor, HER factor 2 and Ki67. The expressions of P receptor, HER factor 2 and Ki67 were closely related. Previous researches found malignancy degree of breast cancer is closely related to its tissue hardness [25]. The UE converts the change of the echo signal movement amplitude before and after compression into a real-time color image according to different elastic coefficients and the degree of deformation of the tissue after being compressed by external force. The tissues with small elastic coefficients and large displacement changes after compression are shown in red. The tissue with large elastic coefficient and small displacement change after compression is displayed in blue. The tissue with medium elastic coefficient is displayed in green. The color of UE imaging indicated the hardness of tissue [26]. Quantification by scoring can accurately reflect the stiffness of tumor tissues. P receptor is induced and secreted by the binding of estrogen to its receptor, which can promote the malignant proliferation of breast cancer tumor cells and increase tissue stiffness [27]. HER factor 2 is an important marker in several malignant tumors. Its overexpression will lead to active tumor cell proliferation, resulting in insufficient energy and oxygen for cell metabolism and stimulating local calcium secretion and calcification in tumors. At the same time, studies have confirmed that overexpression of HER factor 2 can up-regulate the expression of angiogenesis-related factors in breast cells and promote angiogenesis in breast masses and tumor cell proliferation, thereby increasing the mass hardness [28]. This result is consistent with Yin *J* [29]. Ki67 can be expressed in various stages of cell proliferation except for G0 phase of cell quiescence, so its high expression indicates that local cells are in active proliferation phase, in which local cells proliferate rapidly and continue to invade and adhere to the extracellular matrix, resulting in abnormal structure and function of extracellular matrix cohesin. The abnormal extracellular matrix cohesin further promotes the adhesion of the mass to the surrounding tissue [30], which results in low mass elasticity and increase in hardness. The conclusion was in agreement with the research of Veronika et al [31]. Therefore, the expression of P receptor, HER factor 2, and Ki67 can also reflect the stiffness of tumor tissue related to the results of UE.

RETRACTED

This study is a regression study, which may have certain limitations and retrospective bias. In addition, the sample size of the present research is small, and the source of the sample is relatively single. More objective and accurate conclusions need further multi-center and large-sample studies in prospective studies.

## 5. Conclusion

In this study, we explored the correlation of UES with IBC and biological prognostic factors using monofactor analysis, multiple linear regression analysis and ROC curve. The results revealed the UES has a certain diagnostic value for IBC, and is significantly correlated to the expression of P receptor, HER factor 2 and Ki67, which is meaningful for appraising the prognosis of patients with IBC. However, there were some limitations, such as few detection indicators, small samples and so on. Furthermore, multicenter and large-sample investigations in prospective studies were needed to obtain more accurate conclusions.

## Figures and Tables

**Figure 1:** ROC of UES in diagnosis of IBC.

**Figure 2:** ROC of UES used for evaluating the expression of biological prognostic factors in IBC.

**Figure 3:** Ultrasound images of typical case. (a–c) Conventional ultrasound image of breast with solid hypoechoic nodule. The image showed vertical growth, irregular borders, and speckled hyperechoic within. CDFI: perforator blood flow in the mass; PW: arteries with low velocity and high resistance measured spectrum (RI > 0.7). (d) UE image of the same patient (UES 5 points).

**Table 1:** The diagnostic values of UES for IBC.

UES	Pathological diagnosis		Total
	Malignant	Benign	
Malignant	61	2	63
Benign	5	18	23
Total	6 6	20	86
Sensitivity	Specificity	Accuracy	Positive/negative predictive value
92.42%	90.00%	91.86%	96.83%/78.26%

**Table 2:** Univariate analysis of correlation between the UES and the biological prognostic factors of IBC (mean ± SD).

Index	Result	Number of cases	UES (points)	*t* value	*P* value
E receptor	Positive	23	3.95 ± 0.74	1.182	0.242
	Negative	43	4.17 ± 0.71		

P receptor	Positive	38	3.92 ± 0.73	2.620	0.011
	Negative	28	4.37 ± 0.63		

HER factor 2	Positive	42	3.85 ± 0.70	3.313	0.002
	Negative	24	4.42 ± 0.62		

Ki67	Low expression	20	3.67 ± 0.58	4.777	0.000
	High expression	46	4.43 ± 0.69		

RETRACTED

**Table 3:** ROC analysis of the UES used for evaluating the expression of biological prognostic factors in IBC.

Biological prognostic factor	AUC	*P* value	95% CI	Critical value	Sensitivity (%)	Specificity (%)
P receptor	0.704	<0.001	0.600–0.795	4.12	53.1	81.7
HER factor 2	0.763	<0.001	0.663–0.845	4.08	53.1	95.0
Ki67	0.820	<0.001	0.726–0.893	3.95	62.5	95.0

**Table 4:** Multiple linear regression analysis of UES and expression of biological prognostic factors.

Index	*β* value	*t* value	*P* value
P receptor	0.344	1.015	0.004
HER factor 2	0.375	3.838	0.000
Ki67	0.315	2.763	0.007

**Table 5:** Spearman correlation analysis between UES and expression of biological prognostic factors.

Variable	*r* value	*P* value
P Receptor	0.238	0.011
HER factor 2	0.295	0.002
Ki67	0.33 4	0.024

## Data Availability

The simulation experiment data used to support the findings of this study are available from the corresponding author upon request.
